# Registration and Analysis of Acceleration Data to Recognize Physical Activity

**DOI:** 10.1155/2019/9497151

**Published:** 2019-03-03

**Authors:** Marcin Kołodziej, Andrzej Majkowski, Paweł Tarnowski, Remigiusz J. Rak, Dominik Gebert, Dariusz Sawicki

**Affiliations:** Institute of Theory of Electrical Engineering, Measurements and Information Systems, Warsaw University of Technology, Warsaw, Poland

## Abstract

The purpose of the article is to check whether the acceleration signals recorded by a smartphone help identify a user's physical activity type. The experiments were performed using the application installed in a smartphone, which was located on the hip of a subject. Acceleration signals were recorded for five types of physical activities (running, standing, going up the stairs, going down the stairs, and walking) for four users. The statistical parameters of the signal were used to extract features from the acceleration signal. In order to classify the type of activity, the quadratic discriminant analysis (QDA) was used. The accuracy of the user-independent classification for five types of activities was 83%. The accuracy of the user-dependent classification was in the range from 90% to 95%. The presented results indicate that the acceleration signal recorded by the device placed on the hip of a user allows us to effectively distinguish among several types of physical activity.

## 1. Introduction

In today's world, it can be seen that more and more people are beginning to pay attention to their physical activity. A sedentary lifestyle, whether at home or at work, makes caring for our physical condition not just another addition to everyday activities but also a certain duty toward maintaining our health. Currently, the 10,000 steps per day recommended by specialists [1] take an average person just over an hour. Since cardiovascular diseases are now one of the main causes of death, each of us should sacrifice from 20 minutes to 2 hours a day for physical exercises as they help prevent many of these diseases. In the United States, diseases caused by the lack of physical exercises lead to the death of more people than all forms of cancer combined [2]. In view of the above mentioned aspects, newer solutions are emerging in the market that can be used to monitor daily physical activity, and companies producing devices for athletes are primarily involved in this. In addition, devices to monitor the type of activity performed are also available in the market for the average user.

Several researchers have invested a lot of effort to explore different sensing technologies and have proposed a number of methods to recognize human physical activities [3–5]. Researchers constructed various activity recognition systems that utilized accelerometers to infer the body position; accelerometers can provide acceleration and velocity data largely associated with various human physical activities [6–8].

However, having a specialized solution to monitor physical activity is not necessary. A smartphone can be successfully used for this purpose. Almost every smartphone has an accelerometer, also known as an acceleration transducer. As the name suggests, the accelerometer is used to measure the acceleration affecting a given object. An acceleration transducer allows the position of a device in space to be determined and enables the device to be controlled by motion.

The aim of this article is at analyzing the signal from a smartphone accelerometer, in order to use it to identify the user's physical activity type. To collect data, an Android application written in Java programming language was used.

Activity recognition typically consists of three stages. In the first step, the sensor data are divided into segments, typically using the sliding window technique [6, 9]. The next step is to extract features from the segments. Finally, a classifier is trained over these extracted features. The last task is to use the classifier to associate the sensor data with a predefined activity.

In our research, we used the same approach. We tried to answer the following questions:

1. Does the recorded acceleration signal (accelerometer placed on the user's hips) allow several typical physical activities to be distinguished?
2. Does a set of simple statistical features allow you to distinguish between activities effectively?
3. What types of physical activity are the most difficult to distinguish?
4. Is it possible to create a system that recognizes activities based on data collected only from a specific user or it is better to use data from all users (user-dependent vs user-independent classification)?

Answers to these questions will allow you to assess whether there is a chance to develop an application to recognize user activity with just a smartphone. The presented results should be treated as preliminary. In order to fully estimate the effectiveness of the presented activity recognition system, a larger number of users should be tested.

## 2. Materials

The Huawei P10 smartphone equipped with an iNEMO module (LSM6DSM) was used to record the acceleration signals. The LSM6DSM module has a three-axis accelerometer and a gyroscope. The accelerometer can work in ranges ±2 g, ±4 g, ±8 g, and ±16 g. For each person, the phone was placed on the hip, with the display facing the outside (Figure 1). Physical activity was recorded for four people—two men aged 26 and 56 and two women aged 23 and 46. Each person was asked to perform simple physical activities:

- Running (R)
- Standing (S)
- Going up the stairs (U)
- Going down the stairs (D)
- Walking (W)

Each individual user's data were recorded for each activity for several minutes. The acceleration signals were recorded in the three axes, with a sampling frequency *f*s = 50 Hz, and saved in text files. One line of the file corresponded to a single acceleration measurement and contained information about acceleration values in the *x*-, *y*-, and *z*-axes with respect to time. Files containing the recorded signals were analyzed with use of the PC.

## 3. Methods

### 3.1. Signal Processing

At first, the recorded acceleration signals were visually evaluated and fragments of these, associated with the physical activities of interest, were selected. The fragments in which the person had not yet started to perform the given physical activity were removed. It is worth noting that the recorded acceleration signals contain a gravitational component. During experiments, the smartphone can slightly change its position in relation to the original (in the *x-*, *y-*, and *z*-axis). In this way, the gravity component would decompose in various degrees into the acceleration components associated with the *x*, *y*, and *z* coordinate systems. To eliminate this problem, we decided to use the absolute value of the acceleration signal for further analysis. In this way single, independent of the change of the smartphone position, acceleration signal was obtained. The absolute value *A* of the acceleration signals *A*_*X*_, *A*_*Y*_, and *A*_*Z*_ (in the three axes) was calculated. The signal *A*, calculated for each activity, was divided into windows of the width *N*=200 samples (4 seconds). The windows overlapped every *N*/2 samples.

### 3.2. Feature Extraction

A set of features was calculated from each signal window. We decided to use simple statistical features such as energy: VAR, maximum value: MAX, minimum value: MIN, skewness: SK, kurtosis: KU, and quantiles of order 0.025, 0.25, 0.5, 0.75, 0.095: *Q*025, *Q*25, *Q*5, *Q*75, *Q*095, respectively [10]. In this way, a set of 10 features was obtained for each window (trial). The number of trials for each activity type per user was 22. For all types of one-user activity, the number of trials was 110 (5 activities × 22 windows).

### 3.3. Classification

In order to assess the possibility of recognizing user physical activity on the basis of the acceleration signal, the quadratic discriminant analysis (QDA) [11] classifier was implemented. We decided to use the QDA because we assumed that the features do not have to be separated in a linear way. Another advantage is the ease and speed of training such a classifier in comparison with, for example, neural networks.

The 10-CV test was used as a measure of classification accuracy [12]. In the 10-fold cross-validation test, the original set is randomly partitioned into 10 equal sized subsets. Of the 10 subsets, a single subset is retained as the validation data for testing the model, and the remaining nine subsets are used as data for training. The cross-validation process is then repeated 10 times, with each of the 10 subsets used exactly once as the validation data. The 10 results from the folds are then averaged to produce a single estimation [12].

## 4. Results

The results for the accuracy of classification of the five activity classes for individual users are presented in Table 1 (user-dependent classification). A confusion matrix for subject S1 is presented in Table 2.

The presented results indicate satisfactory recognition efficiency. For all subjects (Table 1), the recognition accuracy was 92%. For a classifier that acted in a random manner, the accuracy would be 20%. An example of a confusion matrix for the subject S1 (Table 2) indicates the existence of problems in recognition between the activity of going up the stairs (U) and down the stairs (D).

Next, features from all the subjects were used for training and testing the QDA classifier in the user-independent mode. As in the previous case, the 10 CV test was used. The accuracy of classification of the five types of activity for all users together was 82%. The confusion matrix is presented in Table 3. Also in this case, it turned out that problems were encountered in recognition of the activity of going up the stairs (U) and down the stairs (D). In addition, for some subjects, walking (W) was recognized as going down the stairs (D), and going up the stairs (U) was classified as walking (W).

Tests similar to real conditions were also performed. Furthermore, all trials were divided into 75% for training and 25% for testing. In this case, the classification accuracy was equal to 83%.

## 5. Discussion

Three seconds of the absolute value *A* of acceleration signal recorded for subject S1 is presented in Figure 2. The highest acceleration values, up to 60 m/s^2^, were recorded during running. The smallest accelerations were recorded obviously during the resting status of the user. For walking, we can observe the increases and decreases in acceleration caused by taking each step.

The features for the entire set of acceleration signals recorded for subject S1 were calculated (Table 4). The maximum value of acceleration for going down the stairs (D) was 26 m/s^2^, for running (R) was 83.9 m/s^2^, for rest (S) was 10.6 m/s^2^, for going up the stairs (U) was 27.4 m/s^2^, and for walking (W) was 48.4 m/s^2^.

Histograms of samples of the acceleration signals recorded for different types of activities are presented in Figure 3.  Figure 4 presents the distribution of features of the acceleration signal for subject S1. The presented results indicate that using only energy and the maximum value of the acceleration signal (calculated for a 4-second window), we can effectively separate activity classes. The problem may be the separation of the activity of going up and down the stairs. The features for these signals are very similar to each other.

Calculations were also carried out to select the best set of features. To this end, the Sequential Forward Selection (SFS) algorithm was used [13]. At this stage, the features collected for all subjects were used. The best features, selected in particular stages of the SFS algorithm, and the accuracy of recognition (ACC) obtained for these features are presented in Table 5. The *Q*75 feature turned out to be the best. The best classification accuracy (0.76) was obtained for three features (KU, *Q*25, and *Q*75).

For comparative purposes, short-time Fourier transform analysis of the recorded acceleration signals was performed [14].  Figure 5 presents the spectrogram for the case in which a user was going down the stairs.

You can observe changes in certain frequencies (5, 12, 21, 28, 34, and 42 seconds) to be dominant. Changes are also caused by the “short walk” on flat places between the building's half-floors.

Figure 6 presents a spectrogram for the case in which the subject was running. We can observe a basic frequency and subsequent harmonics, probably related to the frequency of foot strikes on the ground.

High accuracy of physical activities classification (Tables 1–5) prompts consideration of using the described device in real applications. The best approach seems to be training the recognition system for a specific subject (Table 1). The obtained accuracy of classification was in the range of 90–95%. Results for data collected from all subjects (Table 3) were little less accurate. In this case, the classification accuracy for the five classes was 83%. Simple statistical features and the use of one accelerometer allowed satisfactory results to be obtained.

We performed additional experiments to check whether the use of another classifier could improve the accuracy of movement recognition. For this purpose, commonly known classifiers were tested: decision tree, linear discriminant analysis (LDA), support vector machine (SVM) with linear and quadratic kernel, and nearest neighbor classifier 1-NN. The classification results are shown in Table 6. It turned out that the classification accuracy is better by 2% only when using the SVM classifier with quadratic kernel. Slightly worse results were obtained for the LDA classifier, which implements a linear separation of data. Thus, it seems that the use of the QDA classifier was a good solution.

The accuracy of classification obtained by us is consistent with the results of other studies. In [6], the authors recognize different types of activities (2–6 types) using (2–36) sensors. Most often, these activities include standing, walking, bicycling, running, and going upstairs. The obtained classification results have a very large spread of accuracy, from 42% to 96%. In [15], the dependence of the accuracy of classification on the location of the accelerometer on the subject's body was examined. For most activities, the location turned out to be unimportant, and the accuracy of the classification reached over 90%. In [16], the authors presented a system that used many types of sensors in a smartphone (accelerometer, gyroscope, magnetometer, and barometer) to recognize eight types of activities. For all classifiers, using a combination of four sensors performed better than using only the accelerometer. It improves the recognition accuracy by about 10%. In other studies, the possibility of using only one accelerometer to recognize the type of activity was checked. In [17], six types of activities were identified and statistical and frequency features of the signal were used. The best results (93%) were obtained for the decision tree classifier and time-domain and frequency-domain features (94%).

In summary, it is possible to develop a solution to recognize the user's physical activity using only a smartphone located on the hip. Smartphones are easily available and relatively cheap. In connection with the above, the acceleration classification may be used in fitness applications, which monitor user activity. This mechanism can also be used in the audit of employee activity during the working day. In regards to this topic, the above applications are certainly not exhaustive. With the development of technology, newer sensors are available, but the accelerometer will surely continue to be used in detecting activity.

## 6. Conclusion

Acceleration signals were recorded for the five basic types of user's physical activities. Based on the results of the classification obtained, we can answer the questions from the beginning of the article. (1) The accelerometer placed on the user's hip distinguishes between several types of the user's physical activity. (2) Simple statistical features of the acceleration signal are enough to recognize basic activities. (3) From the considered list of five types of activities, the most difficult to distinguish were going up the stairs (U) and down the stairs (D). (4) It is possible to create a system that recognizes activity based on data collected only from a specific subject (user-dependent), and the recognition then is much more accurate, over 90%. It is also possible to train system based on features from all subjects (user-independent), but the accuracy of classification is less, about 83%.

## Figures and Tables

**Figure 1:** The location of the smartphone with the coordinate axes (*X*, *Y*, and *Z*).

**Figure 2:** Acceleration signal obtained for subject S1 for three seconds for the various physical activities.

**Figure 3:** Histograms of samples of the acceleration signals recorded for different types of activities.

**Figure 4:** Distribution graph of the features of the acceleration signal for subject S1 (4-second window).

**Figure 5:** Spectrogram of the acceleration signal while descending the stairs.

**Figure 6:** Spectrogram of the acceleration signal during running.

**Table 1:** Results of the accuracy of classification of five types of physical activity.

Subject	Accuracy
S1	0.95
S3	0.91
S3	0.90
S4	0.92
Mean	0.92

**Table 2:** Confusion matrix for subject S1.

		Predicted class				
		D	R	S	U	W
True class	D	18	0	0	3	0
	R	0	21	0	0	0
	S	0	0	21	0	0
	U	1	0	0	20	0
	W	0	0	0	0	21

**Table 3:** Confusion matrix.

		Predicted class				
		D	R	S	U	W
True class	D	48	0	0	30	6
	R	0	84	0	0	0
	S	0	0	84	0	0
	U	13	0	0	69	2
	W	19	0	0	1	64

**Table 4:** Features calculated for subject S1.

Feature	D	R	S	U	W
VAR	13.7	197.1	0.1	11.4	43.8
MAX	26.0	83.9	10.6	27.4	48.4
MIN	2.2	0.8	8.9	0.9	0.7
SK	0.7	1.8	−0.2	0.3	1.1
KU	3.8	7.1	32.4	4.2	5.8
Q025	3.8	3.3	9.5	3.3	2.3
Q25	8.3	8.9	9.8	8.3	7.1
Q50	9.9	14.4	9.8	10.1	11.8
Q75	12.1	23.4	9.9	12.4	15.1
Q095	6.0	5.2	9.8	6.3	4.0

**Table 5:** The best features: SFS algorithm.

Number of best features	VAR	MAX	MIN	SK	KU	*Q*025	*Q*25	*Q*5	*Q*75	*Q*095	ACC
1									×		0.72
2							×		×		0.75
3					×		×		×		0.76
4				×	×		×		×		0.76
5	×			×	×		×		×		0.76
6	×	×		×	×		×		×		0.76
7	×	×		×	×		×	×	×		0.75
8	×	×		×	×	×	×	×	×		0.75
9	×	×	×	×	×	×	×	×	×		0.74
10	×	×	×	×	×	×	×	×	×	×	0.73

**Table 6:** Comparison of classification results.

Classifier type	Classification accuracy (%)
QDA	82
Decision tree	83
LDA	73
SVM-LINEAR	80
SVM-QUADRATIC	84
1-NN	82

## Data Availability

Data used to support the findings of this study are available from the corresponding author upon request.
